# Effect of Surfosept and Deconex® 53 Disinfectant Agents on the Accuracy and Dimensional Stability of Panasil Dental Impression Materials: An Experimental Study

**DOI:** 10.1155/2021/1248531

**Published:** 2021-10-21

**Authors:** Mostafa Alam, Parviz Amini, Arash Ghaffarpasand, Nasim Khajeh Dalooei, Alireza Hadi, Kamyar Abbasi

**Affiliations:** ^1^Department of Oral & Maxillofacial Surgery, School of Dentistry, Shahid Beheshti University of Medical Sciences, Tehran, Iran; ^2^Department of Prosthodontics, School of Dentistry, Kerman University of Medical Sciences, Kerman, Iran; ^3^Private Practice, Tehran, Iran; ^4^Department of Prosthodontics, School of Dentistry, Shahid Beheshti University of Medical Sciences, Tehran, Iran

## Abstract

**Materials and Methods:**

This in vitro study was performed on 30 dental casts. The samples were divided into one control group and two experimental groups to be disinfected with Surfosept (1%) and Deconex® 53 (2%) using a sequential sampling method (10 per group). The impressions in the experimental groups (i.e., Surfosept and Deconex® 53) were rinsed and dried; then, the disinfectant was sprayed on the impressions and remained for 30 seconds before pouring with stone. In the control group, the impressions were only rinsed and dried and were poured in 10 minutes. Cast dimensions were measured by a profile projector device, and the mean values obtained from the experimental groups were compared with those of the control group.

**Results:**

There were no significant differences among the groups regarding the height of the resulting dies without undercut (*P*=0.62). Moreover, there was no significant difference among the groups regarding the distance between the two dies (*P*=0.77). However, the diameter of the dies with undercut and without undercut was different significantly among the control and experimental groups (*P* < 0.005).

**Conclusion:**

In general, no significant difference was encountered between dimensional stability and accuracy of the dental impressions using Surfosept and Deconex® 53 in this study.

## 1. Introduction

Dental materials are exposed to various pathogenic microorganisms which are potentially harmful [1]. The main source of cross-contamination especially between dental offices and laboratories is due to the contaminated impression trays, dental impression materials, and stone casts [2]. Several methods of disinfection such as chemical disinfection with the immersion method or spray method, microwave, and ultraviolet radiation are used to disinfect the dental impressions and dental casts [3]. Chemical disinfection has remained a common practical approach to eliminate microorganisms, since heat or steam sterilization of impressions and occlusal records cannot be performed due to the risk of distortion [3]. However, as all disinfectant solutions can have remarkable effects on the dimensional changes of impression materials, immersion duration is recommended to be short, i.e., less than 30 minutes [4].

There is invaluable evidence to support the transmission of microorganisms through impression materials [5, 6]. According to the literature, most of the materials used in dental laboratories contain various infectious microorganisms, such as *Streptococci* [7, 8]. Badaró et al. estimated the prevalence of *Streptococci, Staphylococcus aureus, Methicillin-resistant Staphylococcus*, and *Candida* in the impressions taken from the patients' mouths at 100%, 55.6%, 25%, and 9%, respectively [9]. In the current COVID-19 pandemic, proper care should be given to reduce possibility of coronavirus cross-contamination. According to Kampf et al., disinfection with 0.1% sodium hypochlorite or 62–71% ethanol can significantly reduce coronavirus load on surfaces within 1 min exposure time [10]. Therefore, disinfection of dental impressions can remarkably reduce the number of microorganisms.

It is of utmost importance to select the suitable material for disinfection and to identify the potential problems with each approach [11]. Shelf life, solidification, ease of application, low price, robustness, and resistance to different kinds of stress are among suitable characteristics of impression materials [12, 13]. On the other hand, dimensional changes of the impression materials, following the use of disinfectants, are among the main problems in the process of preparation of dental prostheses. Silicones are the most common impression materials used to fabricate fixed dental prosthesis [14]. Recently, the use of addition silicone impressions is escalated due to its high accuracy [3]. Addition-type silicone impression materials with enhanced hydrophilic properties have the potential to show larger dimensional changes after disinfection, compared to conventional condensation-type materials, due to the fact that disinfection solutions may promote water absorption from surrounding environment [15]; however, there is a dearth of research in this regard in the literature. Deconex® 53 is a disinfectant solution, which is commonly used in hospital settings for disinfecting flexible and rigid endoscopes. The recommended concentration of this substance is 1-2% depending on the expected effect, while a maximum of 4% concentration is used in certain circumstances [12]. This solution is composed of alkyl propylene diamine guanidinium diacetate and N-didecyl-N-methyl-poly (oxyethyl) ammonium propionate. Surfosept (Reza Rad Co., Iran) is another alcohol-based disinfectant material which is used for cleaning surfaces and objects. This substance is standardized by the European Medicines Agency (Standards EN 1040). It can also be utilized to disinfect dental instruments. It can be used for eliminating bacteria and viruses, such as influenza A virus subtype H1N1, hepatitis C virus, hepatitis B virus, and human immunodeficiency virus. This solution contains isopropanol, didecyldimethylammonium chloride, ethanol, and other additives [16].

As dental impression material such as elastomeric silicone carries the risk of microbial colonization and infection, of particular concern is the biocompatibility of the disinfection solutions applied on them. Alcohol-based solutions (Surfosept in this study) are found to act as bactericidal, fungicidal, and virucidal against enveloped viruses (e.g., HIV) and have low cytotoxicity to human cells [17].

Also, studies of bacterial resistance to antibacterial agents such as Deconex (a quaternary ammonium salt) have shown a loss of bacterial resistance upon application of them to the surface [18]. The effect of Deconex on the dimensional changes of impression materials has been investigated in some studies; however, there is no study assessing the dimensional changes in the casts disinfected by Surfosept material. As disinfecting dental impressions is necessary, there is a need to investigate different disinfection materials and their effects on the characteristics of impression materials, especially their dimensional changes. Therefore, this study aimed to determine the effect of two substances (i.e., Surfosept and Deconex® 53) on the accuracy and dimensional stability of dental impressions made of addition silicones (i.e., Panasil®).

## 2. Materials and Methods

### 2.1. Metal Bases and Dies

This in vitro experimental study was performed on 30 casts. Samples were divided into one control group and two experimental groups to be disinfected by Surfosept and Deconex® 53 using a sequential sampling method (10 per group). The study included two upper and lower sections simulated based on an intraoral dentate situation (Figure 1). The lower section had a metal base including two stainless steel dies with three degrees taper per each wall. One of the dies was trimmed in a horizontal direction at the cervical region (2 mm) to create an undercut with depth of 1.5 mm and 45 degrees angle. The metal base had four guide bars for placing the upper section in a specified direction. The die base consisted of a metal plate with dimensions of 30 mm width, 60 mm height, and 15 mm length. The upper section, which acted as a custom impression tray, was made of metal base with holes to provide retention for the impression material and to reduce intersection pressure. Additionally, it had 4 holes on 4 sides to hold the base bars. This section had the same dimensions as the lower section but differed in height (12 mm). The die base and the upper and lower sections were made of E.C.N, and the bars and bushes were made of B.O.Z.

### 2.2. Impression

Initially, using the 2-stage method, two units of putty were mixed with two units of accelerator. The mixture was placed in a horse-shoe shape plastic tray, and the impression was taken. Initially, the required space for the wash layer was provided with a 1.5 mm metal spacer. The initial setting time, working time, and total setting time lasted 120, 120, and 240 seconds, respectively, at 32°C.

After the solidification of the impression material, the upper and lower sections were separated and the spacer was removed from the putty material. Light body Panasil® (Kettenbach Co., Germany) was injected on the putty material and around the die, and the impression was taken again. After hardening, the material was separated from the tray following the manufacturer's recommendations. The initial setting time, working time, and the final setting time for the light body material were 150, 60–90, and 240 s, respectively.

### 2.3. Disinfection Process

Deconex® 53 (1%) was sprayed on the impressions for 30 s. In the experimental groups (i.e., Surfosept and Deconex® 53), the impression materials were rinsed and dried after taking impressions. Subsequently, the disinfectant was sprayed on the impressions. The impressions were left in the room temperature for 30 min, for the rebound phenomenon to happen, before pouring them with stone. In the control group, the impressions were washed and dried.

### 2.4. Preparation of BegoStone Samples

In the next stage, the impressions were poured using BegoStone (type IV dental stone) (Wilhelm Herbst Bremen, Germany). According to the guidelines, 50 g of BegoStone was mixed with 10 cc water at 23°C for 30 s, and it was poured into the impressions in three minutes utilizing slow vibration using a dental laboratory vibrator (Silfradent, VIB24, Italy). The casts were separated from the impression after one hour (Figure 2).

### 2.5. A Profile Projector

A profile projector (Tesa Co., Switzerland) with 0.001 mm resolution was utilized to compare the dimensions and geometry of the samples. The profile projector, which is known as an optical comparator, is a shadowgraph device which uses principles of optics for accurate measurement and dimensional inspection of manufactured samples.

### 2.6. Dimensional Measurements

5 variables were specified and examined on cast models. These factors which were measured by the profile projector include the height of the die without undercut (Figure 3(a)), the diameter of the die without undercut (Figure 3(b)), the distance between two dies (Figure 3(c)), the diameter of the die with undercut (Figure 3(d)), and the height of the die with undercut (Figure 3(e)) (Figure 3).

### 2.7. Statistical Analysis

The data were analyzed in the IBM SPSS software (version 21). The three groups were compared in terms of the mean of studied variables. One-way ANOVA was used to compare the groups, and in case of a significant difference, the post hoc test (Tukey test) was used to determine the differences among groups. A *P* value less than 0.05 was considered statistically significant.

## 3. Results

### 3.1. The Mean Height and Diameter Evaluation

The mean height and diameter of the dies with and without undercut and distance between two dies are given in Table 1. The mean height of the dies without undercut was measured at 10.012 mm and 10.014 mm in the Surfosept and Deconex and 10.015 mm in the control group (*P*=0.62). Also, measurements of the mean height of the dies with undercut were found to be the same (*P*=0.62). The mean diameter of the dies without undercut was measured at 8.016 mm and 8.012 mm in the Surfosept and Deconex and 8.035 mm in the control group (*P* < 0.005). Also, the mean diameter of the dies with undercut was measured at 10.04 mm and 10.028 mm in the Surfosept and Deconex and 10.055 mm in the control group (*P* < 0.005). The mean distance between the two dies was measured at 21.739 mm and 21.749 mm in the Surfosept and Deconex and 21.75 mm in the control group (*P*=0.77).

### 3.2. The Mean Difference of Height and Diameter Evaluation

As a result, the height of the dies with or without undercut was the same in the experimental and control groups. The distance between the dies was also calculated to be the similar between the experimental and control groups. Whereas, the diameter of the dies was found to be different, meaning the experimental groups had a lower diameter of the dies, with or without undercut, compared to the control group (*P* < 0.005).  Table 2 summarizes the results obtained from the post hoc test.

## 4. Discussion

This study aimed to determine the effect of two disinfectant materials (i.e., Surfosept and Deconex® 53) on the accuracy and dimensional changes of impression materials and the resulting casts. Among disinfectants, quaternary ammonium salts (Deconex) and alcohol-based solutions (Surfosept) are potent candidates with superior antibacterial properties. Therefore, they are biocompatible materials, which have low cytotoxicity to human cells, and at the same time are environment friendly and may be further developed for home use [18]. The dimensional stability of the impression materials can be influenced by several factors, including the contraction during the polymerization and expansion after immersion in disinfectant solutions [19]. The thermal contraction of addition-type silicone rubber impression materials may lead to a 10–12 *μ*m dimensional change in cylindrical stone casts for every 1 mm increase in impression thickness [20].

Addition silicones (i.e., Panasil®) are the impression materials made of polyvinyl siloxane or vinyl polysiloxane. They have maximum dimensional stability and minimum dimensional changes when exposed to disinfectant materials [19]. The polymerization reaction of these materials helps obtain optimal dimensional stability [16]. Due to the novelty of the addition-type silicone, the type of disinfectant suitable for these materials is not properly specified in the literature. It seems that Deconex® 53 tends to be able to absorb water out of the air, which is consistent to the hydrophilic property of an addition silicone material. However, the use of Deconex® 53 with alginate and polyether should be performed with caution, since eliminating microorganisms in these materials could be compromised [12]. Hiraguchi et al. used addition-type silicones to assess the dimensional changes of impression materials after immersing in glutaraldehyde (2%) and orthophthalaldehyde (0.55%) for 30 min. According to the results of the aforementioned study, no remarkable dimensional changes were observed in casts [20]. This finding was in line with the results obtained from other similar studies [21], in which the use of addition silicone (i.e., Panasil®) was suggested as a suitable impression material.

Comparison of the experimental (i.e., Surfosept and Deconex® 53) and control groups in this study showed that the height of the dies with or without undercut were not significantly different (*P*=0.62). In addition, no significant difference was observed among the groups in terms of the distance between two dies (*P*=0.77). However, there was a significant difference among the groups regarding the diameter of the dies with undercut and the diameter of the dies without undercut (*P* < 0.005). Therefore, no significant difference was found between the experimental and control groups regarding the dimensional changes, except for the diameter of the dies with and without undercut. Based on the obtained results, both Surfosept and Deconex® 53 can be used without significant concern, on the impression materials made of Panasil®.

In a study conducted by Ghasemi et al., Deconex, sodium hypochlorite (25.5%) and Epimax were utilized to disinfect alginate, silicone, and polyether impression materials [12]. According to the results, no significant difference was observed among the impressions in terms of the dimensional changes after disinfection. This finding is consistent with the results obtained from the current study.

Similarly, a study was conducted by Sabouri et al. on 30 impressions to determine the effect of disinfectants on dimensional changes of impression materials. In this study, 20 impressions were disinfected by sodium hypochlorite and acid glutaraldehyde (10 impressions per group) and 10 impressions were considered as a control group. They rinsed impressions with cold water and stored them at room temperature for 30 and 20 min in the disinfected and control groups, respectively. Similar to our study, the height and diameters of the dies and the distance between the dies were measured in three groups. They showed no significant differences between the disinfected and control groups regarding the dimensional changes [22].

In our study, the disinfectant solutions were sprayed on impressions for 30 seconds. Nassar et al. performed a study to determine the effects of disinfectant solutions on the dimensional changes of the impression materials. Four elastomeric impression materials (i.e., Xantopren, Express, Permlastic, and Soft Impregum) were used to compare the effect of immersion time on the dimensional changes of casts made with each of these materials. Dimensional changes were reported in all materials over time, except for immersion periods lower than 20 min [23]. In another study, sodium hypochlorite (25.5%), Deconex, and Sanosil were employed for disinfecting impressions for 8–10 min periods, and the results were acceptable in terms of accuracy and dimensional stability of the material [12].

## 5. Conclusion

The results indicated that the height and the distance between two dies had higher accuracy and dimensional stability following the use of the Surfosept (1%) and Deconex® 53 (2%) disinfecting material. However, in general, no significant difference was noted in terms of influencing the dimensions or accuracy of the impression materials, whether disinfection solutions were used or not.

## Figures and Tables

**Figure 1:** Upper and lower sections simulated based on an intraoral situation.

**Figure 2:** Impression steps: impression obtained from dies (a); poured impression with BegoStone (b); resulting casts (c).

**Figure 3:** The height of the die without undercut (a), the diameter of the die without undercut (b), the distance between two dies (c), the diameter of the die with undercut (d), and the height of the die with undercut (e).

**Table 1:** The mean height and diameter of the die with and without undercut and distance between two dies.

Dimensions	Surfosept		Deconex		Control		*F*	*P* value
	Mean	SD	Mean	SD	Mean	SD		
Height of the die without undercut (mm)	10.012	0.0091	10.014	0.0069	10.015	0.0052	0.43	0.62
Height of the die with undercut (mm)	10.012		10.014		10.015			0.62
Diameter of the die without undercut (mm)	8.016	0.0051	8.012	0.0042	8.035	0.0052	62.723	>0.005
Diameter of the die with undercut (mm)	10.04	0.0047	10.028	0.0042	10.055	0.0085	48.921	>0.005
Distance between two dies	21.739	0.0325	21.749	0.0233	21.75	0.0551	0.258	0.77

**Table 2:** The mean difference of height and diameter of the die with and without undercut and distance between two dies.

Dimensions	Control-Surfosept		*P* value	Control-Deconex		*P* value	Surfosept-Deconex		*P* value
	Mean difference	SD		Mean difference	SD		Mean difference	SD	
Height of the die without undercut (mm)	0.003	0.0032	0.635	0.00100	0.00328	0.95	−0.002	0.0032	0.81
Diameter of the die without undercut (mm)	0.019	0.00219	>0.005	0.023	0.00219	>0.005	0.004	0.00219	0.18
Diameter of the die with undercut (mm)	0.015	0.00274	>0.005	0.027	0.00274	>0.005	0.012	0.00274	>0.005
Distance between two dies	0.0115	0.01759	0.792	0.0012	0.01759	0.99	−0.0103	0.01759	0.82

## Data Availability

The data generated or analyzed are available from the corresponding author upon request.
